# Nutritional and bioactive properties and antioxidant potential of *Amaranthus tricolor*, *A. lividus*, *A viridis,* and *A. spinosus* leafy vegetables

**DOI:** 10.1016/j.heliyon.2024.e30453

**Published:** 2024-04-27

**Authors:** Umakanta Sarker, Shinya Oba, Riaz Ullah, Ahmed Bari, Sezai Ercisli, Sona Skrovankova, Anna Adamkova, Magdalena Zvonkova, Jiri Mlcek

**Affiliations:** a Department of Genetics and Plant Breeding, Faculty of Agriculture, Bangabandhu Sheikh Mujibur Rahman Agricultural University, Gazipur-1706, Bangladesh; b Laboratory of Field Science, Faculty of Applied Biological Sciences, Gifu University, Yanagido 1-1, Gifu 501-1193, Japan; c Department of Pharmacognosy, College of Pharmacy, King Saud University, P.O. Box 2455, Riyadh 11451, Saudi Arabia; d Department of Pharmaceutical Chemistry, College of Pharmacy, King Saud University, Riyadh, Saudi Arabia; e Department of Horticulture, Faculty of Agriculture, Ataturk University, 25240 Erzurum, Turkiye; f Department of Food Analysis and Chemistry, Faculty of Technology, Tomas Bata University in Zlin, Vavreckova 5669, 760 01 Zlin, Czech Republic

**Keywords:** Bioactive compounds, Pigments, Minerals, Protein, DPPH, ABTS^+^, Phenolics, Flavonoids, Weedy and cultivated amaranth, Antioxidant activity

## Abstract

Climate change results in continuous warming of the planet, threatening sustainable crop production around the world. Amaranth is an abiotic stress-tolerant, climate-resilient, C_4_ leafy orphan vegetable that has grown rapidly with great divergence and potential usage. The C_4_ photosynthesis allows amaranth to be grown as a sustainable future food crop across the world. Most amaranth species grow as weeds in many parts of the world, however, a few amaranth species can be also found in cultivated form. Weed species can be used as a folk medicine to relieve pain or reduce fever thanks to their antipyretic and analgesic properties. In this study, nutritional value, bioactive pigments, bioactive compounds content, and radical scavenging potential (RSP) of four weedy and cultivated (WC) amaranth species were evaluated. The highest dry matter, carbohydrate content, ash, content of iron, copper, sodium, boron, molybdenum, zinc, β-carotene and carotenoids, vitamin C, total polyphenols (TP), RSP (DPPH), and RSP (ABTS^+^) was determined in *Amaranthus viridis* (AV). On the other hand, *A. spinosus* (AS) was found to have the highest content of protein, fat, dietary fiber, manganese, molybdenum, and total flavonoids (TF). In *A. tricolor* (AT) species the highest total chlorophyll, chlorophyll *a* and *b*, betaxanthin, betacyanin, and betalain content was determined. *A. lividus* (AL) was evaluated as the highest source of energy. AV and AT accessions are underutilized but promising vegetables due to their bioactive phytochemicals and antioxidants.

## 1 Introduction

Food insecurity and the overall scarcity of calorie intake prevalent mainly in developing countries have led to malnourishment affecting around 795 million people around the world [1]. Among them, approximately 20 million are suffering from concealed hunger on account of mineral and vitamin deficiency [2]. Main foods are considered the key origin of energy, but these sources can be deficient in iron, zinc, iodine, vitamin E, ascorbic acid, and carotenoids [3]. Eating main foods can result in concealed hunger [2]. However, eating main foods including fruits and vegetables on a daily basis as well confirms a robust diet with an equilibrium mineral and vitamin intake [4].

*Amaranthus* leaves comprise more calcium (20 folds), vitamin C (13 folds), iron (7 folds), and beta-carotene (18 folds) in comparison with lettuce [5]. This fast-growing and low-cost vegetable has a C_4_ pathway and multipurpose uses, including growing amaranth as grains ornamentals, or vegetables. Edible fleshy and juvenile aerial parts of amaranth are abundant in protein, digestible fiber, carotenoids, vitamin C, and several elements, such as phosphorus, magnesium, copper, sulfur, calcium, zinc, potassium, sodium, manganese, boron, molybdenum, and iron [[6], [7], [8], [9], [10], [11], [12], [13]]. It also has plentiful colorants, such as betalains, betaxanthins, carotenoids, chlorophylls, and betacyanins [[14], [15], [16], [17], [18], [19]], and bioactives including vitamin C, phenols, their acids, and ﬂavonoids [[20], [21], [22], [23], [24]]. These pigments and phytochemicals have an important ability to quench free radicals, contribute to potential health benefits, and largely impact the food industries [[25], [26], [27]]. These bioactive components can contribute to the prophylaxis and treatment of various ailments, like heart diseases, melanoma, atherosclerosis, emphysema, cataracts, disease of the retina, joint inflammation, and brain degeneration [[28], [29], [30], [31], [32]]. Amaranth species have great adaptability to drought [[33], [34], [35], [36]] and salinity [[37], [38], [39], [40]].

Cultivated species [*A. lividus* L. (AL) *and A. tricolor* L. (AT)] and weedy species [*A. viridis* L. (AV) and *A. spinosus* L. *(*AS)] have spread extensively over the world, including Africa, South East Asia, Australia, the Americas, and Europe. Weedy amaranth and AT are eaten as leafy vegetables (LV) in the early stage. On the other hand, AL is consumed both as an LV in the early stage and curry vegetable (only stem) in the late stage. The edible large barreled fleshy stalks of AL are eaten as popular year-round vegetables up to flowering in Bangladesh, India, and Southeast Asia. WC species have great variability and phenotypic plasticity in Bangladesh, tropical Africa, South East Asia, Australia, the Americas, and Europe [41]. Weedy species are grown like weeds in the crop field, on the roadsides, and on fallow lands. The harvested young twigs, including baby leaves of weedy species, are typically sold on the market for fried, cooked, or steamed vegetables [42,43]. The attractive color, nutritional value, and pleasant taste of amaranth have made it a popular LV in both Asian and global cuisine. Weedy species can be used as a folk medication to alleviate pain and reduce fever because of their antipyretic and analgesic properties. AV has anti-nociceptive, antioxidant, antimicrobial, anti-inflammatory, hepatoprotective, antihyperglycemic, hypolipidemic, antiphytopathogenic, antidiabetic, and anthelmintic activity [42,43]. Both AV and AS can be used in various therapeutic applications including as a diuretic, astringent, emollient, sudorific, or diaphoretic agent, but also as a supportive treatment for conditions such as gonorrhea, hemorrhoids, febrifuge, eczema, galactagogue, earache, bronchitis, burns, boils, wounds, the remedy of snake-bites, internal bleeding, menorrhagia, diarrhea, ulcerated mouths, stomach disorders, nosebleeds, wounds, and dysentery [42,43].

Not many detailed studies have been performed to assess the presence and amount of nutraceuticals, bioactive pigments, chemicals, and RSP in WC amaranth species. Stintzing et al. [44] noted only caffeic and ferulic acids, quercetin, and betacyanins in AS stem*.* However, the research on other species, such as *A. hypochondiacus*, *A. caudatus,* and *A. cruentus* has shown that amaranth leaves contain many times more nutraceuticals, bioactive pigments, phytochemicals, and RSP than the stem [45]. In recent years, we have been studying the chance of using amaranth as a basis of bioactive colorants owing to ample betacyanins, betalains, betaxanthins, and other bioactive chemicals [28,29]. Therefore, in this evaluation, we aim to investigate the nutritive value, bioactive pigments and other bioactive compounds content, and RSPs of WC species. We eventually evaluated the opportunity of the accessions for plentiful bioactive pigments, phytochemicals, nutraceuticals, and antioxidant potential for achieving sufficiency in nutraceuticals and antioxidants.

## 2 Materials and methods

### 2.1 Materials

Four weedy and cultivated amaranth species such as AT, AL, AS, and AV were provided for analysis by the Department of Genetics and Plant Breeding (DGPB). Sixteen accessions (from each species four accessions were selected i. e., accessions AT3, AT4, AT6, and AT10 from *A. tricolor* species; accessions AL3*,* AL6*,* AL8*,* and AL11 from *A. lividus* species; accessions WAS5, WAS7, WAS9, and WAS14 from *A. spinosus* species and accessions WAV2, WAV4, WAV5, and WAV8 from *A. viridis* species) from DGPB based on different agronomic traits, including high yields, antioxidant capacity, and different eco-geographical zones, were chosen. Sixteen accessions of four amaranth species were grown to evaluate bioactive compounds, pigments, nutraceuticals, bioactive phytochemicals, and radical scavenging ability. The seeds of these accessions were obtained from the gene bank of DGPB.

### 2.2 Design and layout

The study was performed using a random design with 3 blocks. Each unit of the study comprises a 1 m^2^ plot succeeding the rows and plants arrangement of 20 and 5 cm, correspondingly. A field layout of the study is presented in Fig. 1.

**Fig. 1:** A field layout of the study showing the placement of genotypes using randomization in 48 experimental units with three replications.

### 2.3 Intercultural practices

At the time of land preparation, compost (10 t/ha) was used. Compost was prepared by piling (1 m height) 1 ton cow dung as the main material and 500 kg rice straw (chopped and prior to composting process these are soaked in the water for 1 d) in a shaded area. The composting procedure lasts for 1 month. Every week, we ensured aeration mixing manually. Water was added to continue the moistness at 50–60 % until the whole process period. A plastic foil was used to cover the pile and protect it from evaporation. We turned it over once a week. Urea, TSP, MP, and gypsum were used at 200, 100, 150, and 30 kg/ha, correspondingly. Plant spacing was upheld ensuing suitable thinning. Weeds were destroyed by means of weeding at consistent breaks. Consistent irrigation was upheld to ensure the satisfactory development of crops. 30 d old leaves were sampled from 25 randomly selected plants.

### 2.4 Reagents and solvent

Reagents: H_2_SO_4_, cesium chloride, HClO_4_, HNO_3_, ABTS^+^, vitamin C, AlCl_3_H_12_O_6_, Trolox, dithiothreitol (DTT), rutin, DPPH, 2, 2-dipyridyl, Folin-Ciocalteu reagent, potassium acetate, standard compounds of pure quercetin, hyperoside, iso-quercetin, myricetin, kaempferol, catechin, apigenin, naringenin, acetic and acid acetonitrile (HPLC grade), potassium persulfate, sodium carbonate, and gallic acid. Solvent: MeOH, hexane, and acetone.

### 2.5 Proximate composition

The fat, fiber, ash, moisture, protein, and gross energy were estimated utilizing the AOAC methods [46]. Nitrogen (N) was estimated using the Micro-Kjeldahl method [33,47]. N was multiplied by 6.25 to measure protein. Protein, ash, moisture, and fat (%) were subtracted from 100 for carbohydrate estimation (g 100 g^−1^ FW).

### 2.6 Mineral composition

The dried leaves (at 70 °C for 24 h) were ground in a mill. Mineral elements were measured from powdered leaves (0.5 g) by subsequent digestion with 40 mL HClO_3_ (70 %), 400 mL HNO_3_ (65 %), and 10 mL H_2_SO_4_ (96 %) [48]. A Hitachi Atomic absorption spectrophotometry (with flame) (Japan) [22,38] was utilized to take the absorbance at prescribed wavelengths for the elements. Macroelements were expressed in mg g^−1^ FW and microelements in μg g^−1^ FW.

### 2.7 Estimation of carotenoids and chlorophylls

Carotenoids and chlorophylls were measured by elicitation of the leaves in C_3_H_6_O (80 %) [33,49]. A Hitachi, spectrophotometer (Japan) was utilized to take the absorbance at 646, 470, and 663 nm. Chlorophylls and carotenoids were measured as mg 100 g^−1^ and total μg g^−1^ of fresh weight.

### 2.8 Betacyanins and betaxanthins content measurement

The leaves were extracted in 80 % methanol containing 50 mM vitamin C. The previously used method was utilized [33,49]. The pigments were estimated by a spectrophotometer at 540 and 475 nm wavelengths. Betacyanins and betaxanthins results were expressed as nanograms of betanin and indicaxanthin equivalent per gram of fresh weight.

### 2.9 β-Carotene

Exactly 0.5 g leaves were thoroughly ground using a mortar and pestle in 10 mL acetone (80 %) and centrifuged at 10,000 rpm for 3–4 min to estimate β-carotene [33,49]. A spectrophotometer (Tokyo, Japan) was utilized to take the absorbance at 510 and 480 nm, respectively. β-carotene was expressed as milligrams of β-carotene per 100 g of fresh leaves.

### 2.10 Vitamin C

DHA and vitamin C were determined using a spectrophotometer. The fresh leaves were pre-incubated using Dithiothreitol (DTT) to reduce dehydroascorbate to ascorbate. The reduction of vitamin C transformed ferric ions into a ferrous ion. 2, 2-dipyridyl transformed into a Fe^2+^ complex due to the reduction of ferrous ions [33,49]. Vitamin C was measured using a spectrophotometer (Hitachi, Japan) by taking the absorbance of complexes at 525 nm. vitamin C was measured in mg per 100 g of fresh weight.

### 2.11 Samples extraction and TP, TF, and RSP determination

In a shady place, the leaves were dried. Both the fresh and dried ground leaves were extracted separately with a mortar and a pestle. Total polyphenols (TP) were estimated from fresh samples, while RSP and total flavonoids (TF) were estimated from dried samples. 10 mL MeOH (90 %) was added to 0.25 g of leaves and the extract was kept in a capped test bottle. Then the bottle was placed at 60 °C in a shaking water bath (Tokyo, Japan). After 1 h, the extract was filtered and stored. The Folin-Ciocalteu reagent [33,50] and AlCl_3_ colorimetric method [33,51] were used to estimate TP and TF. A Hitachi spectrophotometer (Japan) was used to take the absorbance at 760 and 415 nm. TF and TP were expressed as rutin and gallic acid equivalent μg RE g^−1^ DW and μg GAE g^−1^ of FW using standard rutin and gallic acid curves. The diphenyl-picrylhydrazyl (DPPH) radical degradation method and the ABTS^+^ assay method were used to estimate the RSP [33,51,52]. The RSP was measured % of inhibition of DPPH and ABTS^+^ equivalent to the control using following the equation:

(1) RSP(%)=(Ac−As/Ac)×100

where *Ac* is the absorbance of the control [150 μL and 10 μL MeOH for RSP (ABTS), RSP (DPPH)) instead of leaf extract] and *As* is the absorbance of the samples. The results were calculated as μg Trolox equivalent g^−1^ DW.

### 2.12 Samples extraction and determination of phenolic compounds by HPLC and LC-MS

Fresh leaf samples (1 g) were extracted in 10 mL MeOH (80 %) comprising acetic acid (1 %). The mixture was transferred into a capped test tube (50 mL). The test tube was shaken in a Scientiﬁc Industries Inc. shaker (USA) for 15 h at 400 rpm. The extract was ﬁltered using a ﬁlter (0.45 μm MA, USA) and centrifuged at 10,000 rpm for 15 min. The supernatant was used to measure phenolic compounds. All determinations were done in 3 replicates. Shimadzu HPLC (Kyoto, Japan) was used to determine phenolic compounds following the previously described method [16,33,49]. HPLC consisted of a degasser, a binary pump, and a detector. phenolic compounds were separated using a STR ODS-II column (150 × 4.6 mm, 5 μm; Shinwa Chemical Industries, Ltd., Kyoto, Japan). Solvent A and solvent B [acetic acid and acetonitrile 6 % (v/v) in water in water] were pumped at 1 mL/min for 70 min. A gradient program was followed to run the HPLC system with 0–15 % acetonitrile for 45 min, 15–30 % for 15 min, 30–50 % for 5 min, and 50–100 % for 5 min. A column temperature of 35 °C was maintained with an injection volume of 10 μL. The detector was set at 370, 280, and 360 nm. The retention time and UV–VIS spectra were compared to their respective standards for identiﬁcation of the compounds. Phenolic compounds were determined by the mass spectrometry assay method (expressed as μg g^−1^ FW). A mass spectrometer (Tokyo, Japan) was ﬁtted with an Agilent 1100 Series HPLC system and a UV–VIS detector coupled online with an ElectroSpray Ionization (ESI) source to analyze the mass spectrometry with negative ion mode with the column elutes in the range of *m*/*z* 0–1000 and needle voltage at −2000V. A column (STR ODS-II, 150 × 4.6 mm, 5 μm; Kyoto, Japan) was set with a solvent flow rate of 0.7 mL/min at 35 °C for the separation of phenolic compound compounds [52]. Solvent A was 1 % acetic acid and solvent B was acetonitrile. Human metabolites database, CMID, and Metline database were used to identify compounds. Separation was achieved with the initial mobile phase concentration set at 0–15 % B for 45 min, 15–30 % B for 20 min, 30–50 % B for 15 min, and 50–100 % B for 10 min. Extract constituents were identiﬁed by LC-MS-ESI analysis.

### 2.13 Phenolic compound quantiﬁcation

Each phenolic compound was quantified using the respective standards of calibration curves. Nine phenolic compounds were dissolved in MeOH (80 %) as stock solutions to the ﬁnal concentration of 100 mg/mL. The individual phenolic compounds were quantified with external standards using respective standard curves (10, 20, 40, 60, 80, and 100 mg/mL). For identiﬁcation of the phenolic compounds, retention times, co-chromatography of samples, and UV spectral characteristics with commercially available standards were utilized.

### 2.14 Statistical analysis

The mean data of all samples was the mean for each replication. ANOVA was analyzed using Statistix 8 software [[53], [54], [55], [56], [57]]. The Duncan Multiple Range Test was performed to compare means data at a 1 % level of probability. The results were obtainable as the mean ± SD.

## 3 Results and discussion

ANOVA analysis indicated a noteworthy difference for our examined characters. A significant variation in the analysis of variance was found also in agronomic traits of maize [[58], [59], [60], [61]], rice [[62], [63], [64], [65], [66], [67], [68], [69], [70], [71], [72], [73], [74], [75], [76], [77], [78], [79], [80]], okra [[81], [82], [83]], broccoli [84], pulses [[85], [86], [87]], and coconut [88,89] which confirmed our current findings.

### 3.1 Proximate composition

Fig. 2 shows the fat, carbohydrates, moisture, ash, fiber, protein (g 100 g^−1^ FW), and energy (kcal 100 g^−1^ FW) of WC amaranth species. The moisture of WC amaranth species ranged from 81.68 to 86.75. The highest moisture was observed in AT and AS accessions (86.75 and 85.43, respectively). Inversely, the lowest moisture was observed in AV accessions (81.68) and AL accessions (82.96). As lesser moisture corresponds with higher dry mass, AV and AL accessions consisted of 17–18 % dry matter. The findings were corroborative of AT [33] and *Ipomoea batata* leaves [90].

**Fig. 2:** Macronutrient compositions, moisture, fiber, ash (g 100 g^−1^ FW), and energy (kcal) of four weedy and cultivar of amaranth species, (n = 6), Different letters mean statistical significance evaluated by DMRT (P < 0.01), * average of four accessions.

As LVs, leaves of WC amaranth species exhibited high protein content that significantly varied regarding species (5.43–5.88). AS accessions confirmed the highest protein (5.88), which had statistical similarity to AT accessions. Conversely, AL (5.43) and AV (5.44) accessions confirmed the lowest protein. As LVs, WC accessions confirmed high protein. Marginal people and vegetarians in developing countries generally trust amaranth, soybean, and broccoli [[91], [92], [93], [94], [95]] as a basis for protein. The protein of WC amaranth was greatly higher than AT (1.26 %) in earlier investigations [9]. As an LV, WC amaranth species confirmed low-fat which can be eaten as a diet free from cholesterol. The WC amaranth species confirmed noteworthy differences in fat (0.29–0.74). The fat of WC amaranth species confirmed the order: AS > AV > AL = AT. The WC amaranth results conformed with the results of AT [33] and *Ipomoea batata* leaves [90], respectively. They specified that visceral fat covers the physique's tissues controls the function of cells and continues the physique's temperature. The principal origins of essential fats from vegetables are ω-6 and ω-3. Fats make a noteworthy contribution to the digestion, absorption, and transportation of vitamins E, D, A, and K.

The WC amaranth species ensured better carbohydrates with sufficient differences regarding species (2.59–6.78). AV accessions confirmed the highest carbohydrate content (6.78) thereafter AL accessions, while AS accessions confirmed the lowest carbohydrates (2.59) that had statistical similarity to AT accessions. The WC amaranth species predominantly varied pertaining to energy (28.78–52.78). AL accessions confirmed the lowest energy (52.78). Inversely, the lowest energy was confirmed in AS accessions (28.78). The energy of WC amaranth species confirmed the order: AL > AT > AV > AS. AV accessions exhibited the highest ash (6.37). Conversely, AT accessions confirmed the lowest ash (4.50). The ash of WC amaranth species confirmed the order: AV > AL = AS > AT.

Digestible fiber predominantly varied regarding WC amaranth species (8.15–10.76). AS accessions confirmed the highest digestible fiber content (10.76) thereafter AV and AT accessions. Conversely, AL accessions confirmed the lowest digestible fiber content (8.15). Fiber plays a major involvement in the increase of digestibility, cure of constipation, and palatability. Current findings revealed that accessions of AV confirmed the maximum dry matter, carbohydrates, and ash content. AS confirmed the highest protein fat, and digestible fiber, while AL accessions confirmed the highest energy. The protein and digestible fiber of WC species were greater than the protein and digestible fiber of red, green, and stem amaranth [96,97,99]. The dry mass and ash from AT and AL accessions were greater than dry matter. The ash of red, green, and stem amaranth [96,97,99], though the carbohydrates of AT and 10.13039/100011659AL accessions were supported by red, green, weedy, and stem amaranth [[96], [97], [98], [99]]. The fat of weedy amaranth was supported by *A. blitum*, red, green, and stem amaranth [96,97,99,100].

### 3.2 Mineral elements

Fig. 3, Fig. 4 show results of mineral elements, such as macro elements (mg g^−1^ FW) and microelements (μg g^−1^ FW) of WC amaranth species. The WC amaranth species confirmed the better potassium. AV accessions confirmed the highest potassium (6.86), thereafter AS accessions. The lowermost potassium was observed in AL accessions (3.74). Potassium of WC amaranth species confirmed the order: AV > AS > AT > AL. The calcium significantly varied regarding WC amaranth species (2.15–2.68). AS accessions exhibited the highest calcium (2.68). In contrast, AV accessions confirmed the lowermost calcium was observed in (2.15). The calcium of WC amaranth species confirmed the order: AS > AV > AT > AL. WC amaranth species showed noteworthy and good magnesium, while differences were minimal across the species (2.86–3.59 mg g^−1^).

**Fig. 3:** Macroelements (mg g^−1^ FW) of four weedy and cultivar of amaranth species, (n = 6), Dissimilar letters in the bar are significantly varied by DMRT (P < 0.01), * average of four accessions.

**Fig. 4:** Microelements (μg g^−1^ FW) of four weedy and cultivars of amaranth species, (n = 6), dissimilar letters in the bar are significantly varied by DMRT (P < 0.01), * average of four accessions.

AV accessions confirmed the highest magnesium (3.59). Conversely, AS accessions exhibited the lowest magnesium content (2.86). The magnesium content of WC amaranth species confirmed the order: AV > AT > AL > AS. The WC amaranth species revealed prominent variations regarding *species* (0.55–0.93)*.* AV accessions proved the highest phosphorus content (0.93). Conversely, AT accessions confirmed the lowest phosphorus content (0.55). The phosphorus content of WC amaranth species confirmed the order: AV > AS > AL > AT. The WC amaranth species confirmed pronounced variations regarding *species* (0.96–1.62)*.* AV accessions exhibited the highest sulfur content (1.62). Conversely, AT accessions confirmed the lowest sulfur content (0.96). The sulfur content of WC amaranth species is explained in the order: AV > AS > AL > AT. It revealed that different amaranth species confirmed ample potassium (6.86) and magnesium (3.59), phosphorus (0.93), sulfur (1.62), and calcium (2.68) (based on fresh weight). In the amaranth literature, sufficient Ca, Mg, and K were recorded [101]. Ca, Mg, and K of the current study were much more visible compared to *Spinacia oleracea*, *Solanum nigrum*, *Brassica oleracea* var. sabellica, and spider flower. Our results revealed that accessions of AV confirmed the highest magnesium, phosphorus, sulfur, and potassium content. AS accessions confirmed the highest calcium content. The magnesium contents of accessions of WC species were superior to the magnesium of green amaranth [97], while potassium observed in AT accessions and weedy species was greater than the potassium of the previous study [97].

The iron confirmed prominent variations regarding WC amaranth species (12.62–22.13). The highest iron was observed in AV (22.13), while AL accessions confirmed the lowest iron (12.62). The iron of WC amaranth species confirmed the order: AV > AS > AT > AL. It was exposed from our study that preponderant differences were recorded in the manganese of the WC amaranth species (4.24–10.25). The manganese was the highest in AS accessions (10.25), while the lowest manganese was observed in AL accessions (4.24). The manganese of WC amaranth species confirmed the order: AS > AT > AV > AL. The copper confirmed an impressive array of differences in the WC amaranth species (1.25–2.94).

AV accessions confirmed the highest copper (2.94), while AT accessions exerted the lowest copper (1.25). The copper of WC amaranth species confirmed the order: AV > AL > AS > AT. The zinc in the WC species fluctuated meaningfully and distinctly (7.56 in AL accessions to 13.67 in AV accessions). The copper of WC amaranth species confirmed the order: AV > AS > AT > AL. The sodium showed prominent variations regarding WC amaranth species (19.71–29.67). The highest sodium was observed in AV accessions (29.67), while the lowest sodium was observed in AL accessions (19.71). The sodium of WC amaranth species confirmed the order: AV > AS > AT > AL. The molybdenum of the WC amaranth species differed significantly and markedly (0.14 in AT accessions to 0.36 in AV accessions). The molybdenum of WC amaranth species confirmed the order: AV = AS > AL = AT. The boron confirmed prominent variations regarding WC amaranth species (4.42–12.67). The highest boron was observed in AV accessions (12.67), while the lowest boron was observed in AT accessions (4.42). The boron of WC amaranth species confirmed the order: AV > AL > AS > AT. Our results revealed that accessions of AV confirmed the highest iron, copper, sodium, boron, molybdenum, and zinc content. AS accessions confirmed the highest manganese and molybdenum content. WC amaranth species confirmed superior iron and zinc than cassava leaves [102] and beach peas [103]. We noted ample iron (22.13), manganese (10.25), zinc (13.67), sodium (29.67), boron (12.67), and molybdenum (0.36), and copper (2.94) (based on fresh weight) in the WC amaranth species. Similarly, in literature [101] adequate manganese, iron, copper, molybdenum, boron, zinc, and sodium in different species of amaranth were observed. Zinc, iron, manganese, and copper in amaranth were greater than *Spinacia oleracea*, *Solanum nigrum*, *Brassica oleracea* var. sabellica, and spider flower. The iron of the WC species' accessions was superior to green amaranth [73].

### 3.3 Bioactive pigments

Fig. 5 demonstrates bioactive colorants, like chlorophylls (μg g^−1^ FW), carotenoids (mg 100 g^−1^ FW), and betalains (ng g^−1^ FW) of WC amaranth species. Prominent variations in chlorophyll *a* were displayed in WC amaranth species (276.63–492.76). AT established the uppermost chlorophyll *a* (492.76). Inversely, the lowermost chlorophyll *a* (276.63) was displayed in AS accessions. Chlorophyll *a* content of WC amaranth species confirmed the order: AT > AL > AV > AS. The WC amaranth species revealed predominant variances in chlorophyll *b* content (145.23–242.78). AT accessions showed the highest chlorophyll *b* content (242.78). In contrast, AV accessions confirmed the lowest chlorophyll *b* content (145.23). Chlorophyll *b* content of WC amaranth species showed the order: AT > AL > AS > AV. Noteworthy variations in total chlorophyll content were noted in the WC amaranth species (428.17–735.54). AT accessions showed the highest total chlorophyll content (735.54), while AS accessions confirmed the lowest total chlorophyll (428.17). The total chlorophyll of WC amaranth species confirmed the order: AT > AL > AV > AS. We observed notable chlorophyll *a* (492.76), total chlorophyll (735.54), and chlorophyll *b* (242.78) in the WC amaranth species*,* which were superior to the chlorophylls of previous results [104]. Chlorophyll *a*, total chlorophyll, and chlorophyll *b* were much superior to chlorophyll *a, a+b*, and *b* of red, green, and stem amaranth [96,97,99].

**Fig. 5:** Colorant composition of four weedy and cultivar of amaranth species, chlorophyll *a, b,* and total chlorophyll (μg g^−1^ FW), betaxanthins, betalains, betacyanins (ng g^−1^ FW), carotenoids (mg 100 g^−1^ FW); (n = 6), Dissimilar letters in the bar are significantly varied by DMRT (P < 0.01), * average of four accessions.

The WC amaranth species confirmed good betacyanins with noteworthy differences among species (281.77–480.48). AT accessions confirmed the highest betacyanins (480.48). Inversely, AV accessions exhibited the lowest betacyanins (281.77). The betacyanins of WC amaranth species confirmed the order: AT > AL > AS > AV. The WC amaranth species showed good betaxanthins with noteworthy differences among species (250.73–501.87). AT accessions confirmed the highest betaxanthins (501.87). Inversely, AV accessions showed the lowest betaxanthins (250.73). The WC amaranth species confirmed good betalains with noteworthy differences among species (532.50–982.35). The betalains were the highest in AT accessions (982.35). In comparison, the lowest betalains were reported in AV accessions (532.50). The carotenoids showed predominant variability in the WC amaranth species (54.59–86.98). The highest carotenoids were recorded in AV accessions (86.98). Whereas AS accessions confirmed the lowest carotenoids (54.59). Our study confirmed notable chlorophyll *a* (492.76), total chlorophyll (735.54), betacyanins (480.48), chlorophyll *b* (242.78), betaxanthins (501.87), betalains (982.35), and carotenoids (86.98) in the 10.13039/100005484WC amaranth species which were supported by chlorophylls, betalains, and carotenoids of green and red amaranth [104]. Our results revealed that AT accessions confirmed the highest chlorophyll *a*, betacyanins, total chlorophyll, betaxanthins, chlorophyll *b*, and betalains; while AV accessions confirmed the highest carotenoids. Betaxanthins, betacyanins, and betalains in the amaranth were much more noticeable than betaxanthins, betacyanins, and betalains of red, green, and stem amaranth [96,97,99].

### 3.4 Phenolic compounds

*λ*_max_, MS^2^, retention time, the molecular ion, and identiﬁed compounds are shown in Table 1. The isolated phenolic compound values from four weedy and cultivars of amaranth species using LC were associated with representative masses of phenolic compound compounds using respective peaks of the compounds. Nine phenolic compound compounds were identified in four weedy and cultivars of amaranth species, such as quercetin, isoquercetin, hyperoside, rutin, kaempferol, myricetin, apigenin, catechin, and naringenin which confirmed significant differences among four species (Table 1, Table 2). Table 2 shows the detected phenolic compounds in four weedy and cultivars of amaranth species. Both AT and AL confirmed nine compounds albeit myricetin, apigenin, catechin, and naringenin were not detected in AS and AV (Table 2).

**Table 1:** Wavelengths (*λ*_max_), mass spectral data, retention time (Rt), and tentative identiﬁcation of phenolic compounds of four weedy and cultivar of amaranth species.

*λ*_max_ (nm)	MS2 (*m*/*z*)	Rt (min)	Molecular ion [M − H]-(*m*/*z*)	Identity of tentative compounds
370	301.04	7.55	301.0426	Quercetin
360	463.3	54.36	463.3215	Iso-quercetin
360	463.5	53.35	463.4621	Hyperoside
360	609.3	53.36	609.3698	Rutin
370	593.3	17.84	593.5312	kaempferol
370	626.2	4.58	626.1882	Myricetin
370	270.3	15.47	270.3432	Apigenin
280	290.2	23.91	290.2287	Catechin
280	271.16	26.74	271.0812	Naringenin

**Table 2:** Phenolic compounds (μg g^−1^ FW) of four weedy and cultivars of amaranth species.

Phenolic compound group	Flavonols						Flavones	Flavanols	Flavanones
*A.* spp.	Quercetin	Iso-quercetin	Hyperoside	Rutin	Kaempferol	Myricetin	Apigenin	Catechin	Naringenin
*A. tricolor*^a^	6.52 ± 0.06a	6.88 ± 0.05a	2.45 ± 0.02a	9.72 ± 0.06a	4.42 ± 0.03a	4.28 ± 0.02a	3.38 ± 0.03a	1.32 ± 0.02b	2.84 ± 0.02a
*A. lividus*^a^	5.35 ± 0.08b	4.75 ± 0.04b	1.52 ± 0.02b	8.46 ± 0.07b	2.26 ± 0.03b	3.14 ± 0.03b	2.42 ± 0.02b	2.27 ± 0.01a	2.24 ± 0.02b
*A. viridis*^a^	4.44 ± 0.06c	4.96 ± 0.03b	1.34 ± 0.01b	6.38 ± 0.08d	4.52 ± 0.02a	nd	nd	nd	nd
*A. spinosus*^a^	3.56 ± 0.07d	3.66 ± 0.03c	2.38 ± 0.02a	7.75 ± 0.08c	2.34 ± 0.02b	nd	nd	nd	nd

Dissimilar letters in the bar are significantly varied by DMRT; nd, not detected; (n = 3); (*P* < 0.01).

a average of four accessions.

Among four main groups of phenolic compounds, the most identiﬁed preponderant compounds in four weedy and cultivar of amaranth species were observed in the order: ﬂavonols > ﬂavones > ﬂavanones > ﬂavanols (Table 2). Except for catechin, AT confirmed the highest quercetin, isoquercetin, hyperoside, rutin, kaempferol, myricetin, apigenin, and naringenin. Similarly, AL confirmed the highest catechin, and both AT and AS confirmed the highest hyperoside. Inversely, AT confirmed the lowest catechin, AV confirmed the lowest quercetin, AS confirmed the lowest rutin, and AL confirmed the lowest isoquercetin, hyperoside, kaempferol, myricetin, apigenin, and naringenin. Among ﬂavonols, ample rutin, quercetin, and isoquercetin among four amaranth species. Quercetin, isoquercetin, hyperoside, rutin, kaempferol, myricetin, apigenin, catechin, and naringenin of four amaranth species diverse from 3.56 to 6.52, 3.66 to 6.88, 1.34 to 2.45, 6.38 to 9.72, 2.26 to 4.52, 3.14 to 4.28, 2.42 to 3.38, 1.32 to 2.27, and 2.24–2.84 μg g^−1^ FW, respectively (Table 2). Weedy species can be used as a folk medication to alleviate pain and reduce fever because of their antipyretic and analgesic properties. AV has anti-nociceptive, antioxidant, antimicrobial, anti-inflammatory, hepatoprotective, antihyperglycemic, hypolipidemic, antiphytopathogenic, antidiabetic, and anthelmintic activity [42,43]. Both AV and AS can be used in various therapeutic applications including as a diuretic, astringent, emollient, sudorific, or diaphoretic agent, but also as a supportive treatment for conditions such as gonorrhea, hemorrhoids, febrifuge, eczema, galactagogue, earache, bronchitis, burns, boils, wounds, the remedy of snake-bites, internal bleeding, menorrhagia, diarrhea, ulcerated mouths, stomach disorders, nosebleeds, wounds, and dysentery [42,43].

### 3.5 Bioactive components and RSP

TP (μg g^−1^ FW), β-carotene (mg 100 g^−1^ FW), total flavonoids (TF, μg g^−1^ DW), vitamin C (mg 100 g^−1^ FW), and RSP (μg g^−1^ DW) of four weedy and cultivar of amaranth species are presented in Fig. 6.

**Fig. 6:** Phytochemicals and RSP of four weedy and cultivars of amaranth species, β-carotene and ascorbic acid (mg 100 g^−1^ FW), TP (μg GE g^−1^ FW), TF (μg RE g^−1^ DW) RSP (ABTS^+^ and DPPH) (μg TE g^−1^ DW); (n = 6), dissimilar letters in the bars signiﬁcantly differed by DMRT (P < 0.01), * average of four accessions.

The noteworthy differences were observed in the β-carotene of WC amaranth species (46.67 in AS accessions to 62.88 in AV accessions). The β-carotene content of WC amaranth species confirmed the order: AV > AT > AS > AL. The WC amaranth species revealed prominent vitamin C variations (46.77–106.21). Vitamin C was the highest in AV accessions (106.21) and the lowest in AS accessions (46.77).

The vitamin C of WC amaranth species confirmed the order: AV > AL > AT > AS. Marked and noteworthy differences were observed in the TP of WC amaranth species (21.30–43.41). AV accessions confirmed the highest TP content (43.41). While AL accessions confirmed the lowest TP (21.30). The TP of WC amaranth species confirmed the order: AV > AT > AS > AL. The WC amaranth species showed high TF with noteworthy differences among species (149.91–179.05). AS accessions confirmed the highest TF (179.05 μg g^−1^). Whereas AL accessions confirmed the lowest TF (149.91). The TF of WC amaranth species confirmed the order: AS > AV > AT > AL. The WC amaranth species established strong RSP (ABTS^+^ and DPPH) among species. AV accessions exhibited the highest DPPH and ABTS^+^ RSP (35.46, 68.43). Inversely, the lowest RSP (ABTS^+^ and DPPH) were documented in AL accessions (25.06, 46.98), which valid the quantification of two different antioxidant capacity methods. In this investigation, TP (43.41), TF (179.05), RSP (DPPH) (35.46), and RSP (ABTS^+^) (68.45) measured in amaranth were greater than previous findings [104]. The carotenoids in amaranth were larger than previous findings [97,99]. The β-carotene, RSP (DPPH), vitamin C, TF, and RSP (ABTS^+^) in this investigation were greater than the β-carotene, RSP (DPPH), vitamin C, TF, and RSP (ABTS^+^) of previous findings [[96], [97], [98], [99]]. The TP was greater than the TP of green amaranth [97]. The WC amaranth species confirmed high antioxidants, flavonoids, and phenolics with substantial vitamins, pigments, and nutrients. These genotypes can be selected as desirable high-yielding cultivars comprising satisfactory antioxidants and apposite for extraction juice. AV accessions confirmed the highest RSP (DPPH), β-carotene, TP, RSP (ABTS^+^), and vitamin C. In contrast, AS accessions confirmed the highest TF.

### 3.6 The correlation studies

The **c**orrelation of bioactive colorants, RSP (DPPH), β-carotene, TP, AsA, TF, and RSP (ABTS^+^) of the WC amaranth species are shown in Table 3. The relationship of bioactive pigments, β-carotene, TP, AsA, TF, RSP (DPPH), and RSP (ABTS^+^) of the WC amaranth species confirmed exciting results. Except for carotenoids, all bioactive pigments positively and significantly correlated with TP, RSP (DPPH), TF, and RSP (ABTS^+^). It specified that the upsurge in TP, RSP (DPPH), TF, and RSP (ABTS^+^) was directly associated with the augmentation of betaxanthins, betacyanins, chlorophylls, and betalains or vice versa. It destined, except for carotenoids, all bioactive pigments confirmed good RSP. β-Carotene, carotenoids, and vitamin C were positively and significantly associated with each other. Similarly, β-carotene, carotenoids, and vitamin C confirmed noteworthy positive relationships with TP, RSP (DPPH and ABTS^+^), and TF although they confirmed negative and nonsignificant relationships among bioactive pigments. In the preceding studies of amaranth [[33], [34], [35], [36], [37]], there were observed a similar trend too. The positive and significant correlations of β-carotene, carotenoids, vitamin C, RSP (DPPH) and RSP (ABTS^+^), TF, and TP suggest that carotenoids, TP, β-carotene, vitamin C, and TF confirmed strong RSP [105,106]. The validation of RSP of the WC amaranth species by two different methods of RSP measurements was confirmed with significant positive associations between RSP of DPPH and RSP of ABTS^+^. Bioactive pigments and phytochemicals including β-carotene, TP, TF, and vitamin C confirmed a strong RSP, as these components confirmed noteworthy associations with both RSP (DPPH and ABTS^+^). All bioactive pigments, β-carotene, carotenoids, TF, TP, and vitamin C carry a dynamic role in the RSP of the WC amaranth species as these compounds confirmed intense RSP.

**Table 3:** The correlation coefficient for pigments, phytochemicals, and RSP in four weedy and cultivars of amaranth species.

	BX	BL	Ch *a*	Ch *b*	T. Ch	CA	BCA	AsA	TP	TF	RSP (DPPH)	RSP (ABTS^+^)
BC	0.98**	0.97**	0.99**	0.98**	0.97**	0.45	0.38	0.21	0.78**	0.66*	0.68*	0.67*
BX		0.98**	0.98**	0.96**	0.99**	0.37	0.26	0.14	0.68*	0.67*	0.64*	0.63*
BL			0.96**	0.94**	0.98**	0.36	0.32	0.18	0.74**	0.63*	0.66*	0.78**
Ch *a*				0.93**	0.98**	−0.18	−0.12	0.15	0.76**	0.62*	0.83**	0.75**
Ch *b*					0.96**	−0.25	−0.23	0.16	0.78**	0.78**	0.64*	0.82**
T. Ch						−0.06	−0.17	0.22	0.77**	0.77**	0.62*	0.64*
CA							0.82**	0.83**	0.86**	0.87**	0.97**	0.96**
BCA								0.75**	0.84**	0.94**	0.63*	0.67*
AsA									0.79**	0.88**	0.78**	0.88**
TP										0.76**	0.86**	0.86**
TF											0.62*	0.76**
RSP (DPPH)												0.96**

BC, Betacyanins; BX, Betaxanthins; BL, Betalains; Ch *a*, Chlorophyll *a*; Ch *b*, Chlorophyll *b*; T. Ch, Total chlorophyll; CA, Carotenoids; BCA, β-carotene; AsA, Ascorbic acid; TP, total polyphenols; total flavonoids; RSP (DPPH), RSP (ABTS^+^); *,**significant at 5 % and 1 % level, (n = 6).

## 4 Conclusions

The WC amaranth species as an LV confirmed abundant sources of magnesium, phosphorus, potassium, sulfur, calcium, iron, boron, manganese, molybdenum, copper, sodium, zinc, protein, digestible fiber, and carbohydrates. It is an outstanding basis for bioactive colorants and bioactive phytonutrients, such as β-carotene, AsA, phenolics, flavonoids, and other antioxidants. The results revealed that AV accessions confirmed the highest dry matter, ash, content of iron, copper, sodium, boron, molybdenum, zinc, carbohydrates, carotenoids, β-carotene, AsA, TP, RSP (DPPH), and RSP (ABTS^+^). AS accessions confirmed the highest protein, fat, digestible fiber, manganese, molybdenum, and TF content. AL accessions were evaluated with the highest energy. AT accessions confirmed the maximum chlorophyll *a*, betaxanthins, total chlorophyll, betalains, chlorophyll *b*, and betacyanins content. Nine phenolic compound compounds were identified in four weedy and cultivars of amaranth species, such as quercetin, isoquercetin, hyperoside, rutin, kaempferol, myricetin, apigenin, catechin, and naringenin. Both AT and AL confirmed nine compounds albeit myricetin, apigenin, catechin, and naringenin were not detected in AS and AV. The most dominant compounds identiﬁed in four weedy and cultivar amaranth species were displayed in the order: ﬂavonols > ﬂavones > ﬂavanones > ﬂavanols. AT confirmed the highest quercetin, isoquercetin, hyperoside, rutin, kaempferol, myricetin, apigenin, and naringenin content, and AL confirmed the highest catechin quantity. Among ﬂavonols, ample rutin, quercetin, and isoquercetin were detected in four weedy and cultivars of amaranth species. The relationship revealed that bioactive colorants and phytonutrients of AT and AV confirmed good RSP (DPPH and ABTS^+^). AV and AT accessions are underutilized but promising vegetables. Its enormous bioactive phytochemicals and antioxidants make it possible to cultivate as preferable cultivars for leafy vegetables. Leaves could be utilized for everyday diets such as leafy vegetables (boiled), fresh salad, and other culinary dishes. On the basis of its nutritious status, it can be equivalent to *Spinacea oleracea* and could be produced year-round during summer, with gaps in vegetables. AV and AT accessions also could be utilized as a possible origin of bioactive colorants, bioactive phytochemicals, and antioxidants to achieve sufficiency in nutrients and antioxidants.

## Data availability statement

Data recorded in the current study are available in all Tables and Figures of the manuscript.

## CRediT authorship contribution statement

**Umakanta Sarker:** Writing – review & editing, Writing – original draft, Validation, Software, Resources, Methodology, Investigation, Formal analysis, Data curation, Conceptualization. **Shinya Oba:** Writing – review & editing, Validation. **Riaz Ullah:** Writing – review & editing, Validation. **Ahmed Bari:** Writing – review & editing, Validation. **Sezai Ercisli:** Writing – review & editing, Validation. **Sona Skrovankova:** Writing – review & editing, Validation. **Anna Adamkova:** Writing – review & editing, Validation. **Magdalena Zvonkova:** Writing – original draft, Validation. **Jiri Mlcek:** Writing – review & editing, Validation.

## Declaration of competing interest

The authors declare that they have no known competing financial interests or personal relationships that could have appeared to influence the work reported in this paper.
